# Construction of Pulmonary Nodule CT Radiomics Random Forest Model Based on Artificial Intelligence Software for STAS Evaluation of Stage IA Lung Adenocarcinoma

**DOI:** 10.1155/2022/2173412

**Published:** 2022-08-28

**Authors:** Qian Liu, Wanyin Qi, Yanping Wu, Yingjun Zhou, Zhiwei Huang

**Affiliations:** ^1^Department of Radiology, The Affiliated Hospital of Southwest Medical University, Luzhou, China; ^2^Department of Radiology, Xiangtan Central Hospital, Xiangtan, China; ^3^School of Medical Information and Engineering, Southwest Medical University, Luzhou, China

## Abstract

**Objective:**

Spread through air space (STAS) is an invasive characterization of lung adenocarcinoma and is regarded as a risk factor for poor prognosis. The aim of this study is to develop a random forest model for preoperative prediction of spread through air spaces (STAS) in stage IA lung adenocarcinoma.

**Methods:**

92 patients with stage IA lung adenocarcinoma, who underwent computed tomography (CT) scan and surgical resection, were retrospectively reviewed. Each pulmonary nodule was automatically segmented by artificial intelligence (AI) software, and its CT-based radiomics were extracted. All patients were pathologically classified into STAS-negative and STAS-positive cohorts; then, clinical pathological and CT-based radiomics were compared between the two cohorts. Finally, a prediction model for evaluating STAS status in stage IA lung adenocarcinoma was established by a random forest model.

**Results:**

Among 92 patients with stage IA lung adenocarcinoma, STAS positive was identified in 19 patients. The random forest classification model identified predictive features, including CT maximum value, consolidation to tumor ratio (CTR), 3D diameter, CT mean value, entropy, and CT minimum value. The misclassification rate of the random forest model is only 7.69%.

**Conclusion:**

The risk factors of STAS in stage IA lung adenocarcinoma can be effectively identified based on the random forest model, and the hierarchical management of characteristic risk can be effectively realized. A random forest model for predicting STAS in IA lung adenocarcinoma is simple and practical.

## 1. Introduction

With the widespread development of low-dose CT examinations, although the screening rate and surgical opportunities for early-stage lung cancer have increased significantly, lung cancer-related mortality still ranks first among all malignant tumors [1]. Lung adenocarcinoma, the primary pathological type of lung cancer, is often manifested as ground-glass nodules on CT in the early stage and can be divided into pure ground-glass nodules and subsolid nodules according to the presence of solid components [2]. The spread through air spaces (STAS) of lung cancer was newly confirmed by the WHO in 2015 and was defined as the presence of tumor cells in the surrounding alveolar space outside the primary focus of lung cancer [3]. It is the fourth metastasis mode after lymphatic metastasis, blood metastasis, and local direct metastasis. STAS has attracted much attention because it can significantly increase the postoperative recurrence rate of early lung cancer [4]. If STAS is present in postoperative pathology of early lung cancer, it is in the category of invasive adenocarcinoma. In other words, adenocarcinoma in situ and microinvasive adenocarcinoma do not present STAS [5]. Among the many risk factors affecting the poor prognosis of the stage IA surgery on early lung cancer, in addition to pleural invasion and vascular invasion, STAS is gradually gaining attention [6]. Both are regarded as indicators of the aggressiveness of early-stage lung cancer. Studies in recent years have shown that STAS is also closely associated with occult lymph node metastasis in stage IA lung adenocarcinoma [7]. In addition, it also significantly increases the risk of recurrence after sublobectomy [8]. After sublobar resection of lung cancer patients, their postoperative recurrence-free survival (RFS) time and overall survival (OS) time were significantly reduced, while when receiving lobectomy, STAS had no significant correlation with RFS and OS. Therefore, accurate imaging diagnosis of STAS for stage IA lung adenocarcinoma before surgery has important reference value for the formulation of surgical scope and evaluation of prognosis.

The previous literature [9] has made a preliminary summary of the imaging manifestations of STAS in lung cancer, including the largest lesion diameter, abnormal bronchial gas phase, the proportion of solid components, and the blurred ground-glass border around subsolid lesions. CT radionics can extract high-throughput texture phenotypes of lung nodules, quantify their imaging features, and establish an objective prediction model for STAS in stage IA lung adenocarcinoma [10]. However, in this study, the extraction of CT texture signs of pulmonary nodules used manual layer-by-layer delineation, which was cumbersome to operate, with significant accumulated errors and poor consistency [11]. It failed to focus on early-stage IA lung adenocarcinoma for further research. With the widespread application of artificial intelligence technology in the screening and diagnosing of lung diseases, the automatic identification and segmentation of pulmonary nodules can be realized based on deep learning algorithms, and its CT texture features can be further extracted [12]. In this study, a random forest model was constructed based on CT texture omics of lung nodules to provide objective and convenient diagnostic ideas for the preoperative diagnosis of STAS in stage IA lung adenocarcinoma.

## 2. Materials and Methods

### 2.1. Case Enrollment

A retrospective analysis was performed on patients with stage IA lung adenocarcinoma who underwent surgical resection in the Affiliated Hospital of Southwest Medical University from January 2017 to June 2021. The hospital ethics committee approved this study. Inclusion criteria for this study is as follows: (1) the patients underwent surgical resection in this medical institution, and the surgical methods were lobectomy, segmental resection, or wedge resection. (2) The surgical and pathological results confirmed lung adenocarcinoma, and the STAS status was recorded. (3) The interval between preoperative CT scan and operation time should not exceed 2 weeks. Exclusion criteria is as follows: (1) interference from other lesions around pulmonary nodules, such as inflammation, atelectasis, and pleural effusion, which limited the identification and segmentation of lesions by artificial intelligence software; (2) combined with other malignant tumors; and (3) partial absence of imaging data or pathological data, poor image quality, etc.

### 2.2. CT Scan and Image Acquisition

The Shanghai United Imaging uCT550 multislice spiral was used for scanning, and the scanning field included the lung apex to the lung base. The scanning parameters are as follows: tube voltage is 120 kV, tube current is 100-150 mA, and the pitch is 1.375-1.5 mm. After scanning, the postprocessing reconstructed slice thickness is 0.625 mm-1.25 mm using standard algorithms. The scanned CT image samples are shown in Figure 1.

### 2.3. Automatic Recognition and Texture Extraction of Pulmonary Nodules

The scanned images are compressed and packaged in DICOM format and exported to the lung nodule artificial intelligence system. The system automatically identifies and extracts CT texture omics parameters of the lesions based on the artificial intelligence system of lung nodules, as shown in Figure 2. CT texture parameters are recorded and extracted by artificial intelligence software of lung nodules, including maximum CT value, minimum CT value, mean CT value, kurtosis, skewness, maximum section area, superficial area, 3D longest diameter, 2D average diameter, compactness, sphericity, and entropy.

Clinical pathological data were collected through the electronic medical record system. The main contents included the age, gender, surgical method, histological type, vascular invasion, nerve invasion, pleural invasion, lymph node metastasis, and STAS. According to the 2015 WHO classification of lung cancer, STAS positive was defined according to clusters, solid nests, or single cells scattered within the airspace outside the boundary of the primary tumor, as shown in Figure 3.

### 2.4. Statistical Analysis

Statistical analysis was performed using RStudio 3.5.1. The software package “Compare Groups” performed univariate analysis on the clinical imaging data of STAS-positive and STAS-negative groups of stage IA lung adenocarcinoma.

The software package “Random Forest” was used to construct a random forest model for the preoperative clinical imaging data. The steps were as follows: (1) random replacement sampling (bagging method, *K* tree value default 500 times) was performed in the training set, and candidate features were extracted to construct a classification tree. Each extraction did not include an average of 36.8% of the original data, that is, out-of-bag (OOB), and used OOB as the test sample. According to the voting results of the classification tree, the classification results of candidate features were determined to form the random forest classification, and OOB was used to test the generalization ability of the model. (2) The Gini coefficient is used to calculate the optimal separation method of each feature for each node in the classification tree. The more the Gini value decreases, the more important the feature becomes [13]. Finally, the diagnostic efficiency of the random forest model is calculated by confusion matrix.

## 3. Experimental Results

### 3.1. Correlation Analysis between STAS and Pathological Results

In this study, 92 patients with stage IA lung adenocarcinoma were collected. The pathological results were divided into 19 cases with STAS positive and 72 cases with STAS negative. This study found that in the postoperative pathological results, histological type, vascular invasion, and lymph node metastasis were closely related to STAS (all *P* < 0.05). In the STAS -positive group, there were more dominant types of acinar composition, papillary, and micropapillary types. In addition, the incidence of vascular invasion and lymph node metastasis was higher. The correlation analysis between STAS and pathological results of stage IA lung adenocarcinoma is shown in Table 1.

### 3.2. Comparison of Preoperative Clinical Imaging Data

Compared with the STAS-negative group, maximum CT value, minimum CT value, average CT value, variance of CT value, maximum area, surface area, 3D length diameter, volume, consolidation to tumor ratio (CTR), and entropy value of the STAS-positive group were greater. In addition, sphericity, compactness, and skewness were lower (all *P* < 0.05). There were no significant differences in age, gender, kurtosis, and position (all *P* > 0.05). The comparison results are shown in Table 2.

### 3.3. Identification of STAS in Stage IA Lung Adenocarcinoma Based on Random Forest

When the random forest method is used to take the default value of *K* trees as 500, the OOB of the model is 7.61%, as shown in Figure 4. The importance of features was ranked by decreasing the mean Gini value, namely, CT maximum, solid ratio, CTR, 3D long axis, CT mean, entropy, and CT minimum, as shown in Figure 5. Through the confusion matrix, it is calculated that the misclassification rate of the random forest model is only 7.69%. It was observed that from the features of CT maximum value, solid ratio, CTR, 3D long diameter, CT average value, entropy, and CT minimum value, the average Gini value of other features did not decrease significantly.

## 4. Discussion

STAS is a significant risk factor for poor postoperative prognosis of stage IA lung adenocarcinoma. This study found that the STAS-positive group had relatively more solid-based and micropapillary-based types in the postoperative pathological results, and these pathological types had a better prognosis. In addition, the incidence of vascular invasion and lymph node metastasis was higher. It can be seen that STAS is an essential indicator for evaluating the aggressiveness of early lung adenocarcinoma, and stage IA lung adenocarcinoma with STAS has a higher degree of malignancy, which is consistent with previous studies. In previous studies, morphological parameters of pulmonary nodules, such as the largest diameter of the lesion, abnormal bronchial gas phase, the proportion of solid components, and blurred ground-glass boundaries around subsolid lesions, were used to evaluate STAS by routine preoperative imaging. It is peculiar and largely depends on the clinical experience of the radiologist. Therefore, it is necessary to deeply mine the imaging features of stage IA lung adenocarcinoma and explore a predictive model with higher diagnostic efficiency and more logical diagnosis ideas.

This study can automatically identify stage IA lung adenocarcinoma lesions and extract their CT texture omics features based on artificial intelligence software for lung nodules. In addition, after obtaining the CT texture parameters of pulmonary nodules, this study used the random forest model to reduce the dimensionality of the clinical image data, and the misclassification rate of the random forest model was only 7.69%. The random forest model is a constitutive machine learning method. Based on the sampling of sample variables, many decision trees are generated to indicate the accuracy of the classification. The OOB error can be obtained by comparing the fundamental categories of the model, and the relative importance of the variables can be calculated. And then, the risk classification is finished [14]. The model in this study finally identified CT maximum value, solid ratio, CTR, 3D long diameter, CT mean value, entropy, and CT minimum value as predictive features of STAS status.

For subsolid pulmonary nodules, the pathological invasiveness depends on the CTR and the size of the lesion [15]. On the other hand, CTR is also an important indicator of various malignant biological characteristics of subsolid nodules. Moreover, OS are closely related. This study also found that higher CT maximum, minimum, and mean values were associated with STAS. Previous studies have pointed out that CT maximum, minimum, and mean values can indicate the pathological infiltration capacity of pulmonary nodules, so it can also evaluate the STAS and other malignancies of pulmonary nodules [16]. The entropy value describes the complexity and irregularity of the lesion composition, reflecting the heterogeneity within the nodule; the higher entropy value of STAS positive corresponds to its biological behavior, such as a greater degree of malignancy and a higher heterogeneity [17]. Finally, in this study, the diagnostic efficiency of the random forest model was analyzed, and its misclassification rate was only 7.69%. It can be seen that the model has great potential for clinical application.

## 5. Conclusion

In this study, the artificial intelligence software of pulmonary nodules can automatically identify, segment, and extract CT texture signs of lesions and mine more quantitative parameters of CT images, which has high diagnostic efficiency. It can be seen that the CT radiomics model based on random forest may become a good tool for preoperative prediction of STAS, which is helpful for surgeons' surgical selection. There are certain limitations in this study. This study is a single-center, retrospective study with a small sample size and failed to conduct a multicenter study, so the results may have selection bias. The dimensionality reduction of various clinical imaging data and radionics parameters before cancer surgery was carried out, but the prediction factors such as molecular biology and genotype were not included, which may limit the generalization ability of the model.

## Figures and Tables

**Figure 1:** CT image samples of pulmonary nodules.

**Figure 2:** Study design process.

**Figure 3:** HE staining (×100) showing STAS (marked by an asterisk).

**Figure 4:** Curves of different classification error rates and OBB classification error rates of the random forest model.

**Figure 5:** Ranking model feature importance by decreasing the average Gini value.

**Table 1:** Postoperative pathological features of stage IA lung adenocarcinoma.

Parameter	STAS negative (*N* = 73)	STAS positive (*N* = 19)	*P* value
Surgery			0.106
Lobectomy or pneumonectomy	25 (34.2%)	11 (57.9%)	
Sublobar resection	48 (65.8%)	8 (42.1%)	
Histologic subtypes			0.020
Papillary	22 (30.1%)	4 (21.1%)	
Solid	3 (4.11%)	3 (15.8%)	
Lepidic	23 (31.5%)	2 (10.5%)	
Micropapillary	3 (4.11%)	4 (21.1%)	
Acinar	22 (30.1%)	6 (31.6%)	
Lymphovascular invasion			0.005
Absent	69 (94.5%)	13 (68.4%)	
Present	4 (5.48%)	6 (31.6%)	
Perineural invasion			0.355
Absent	68 (93.2%)	16 (84.2%)	
Present	5 (6.85%)	3 (15.8%)	
Pleural invasion			0.133
Absent	65 (89.0%)	14 (73.7%)	
Present	8 (11.0%)	5 (26.3%)	
Lymph node metastasis			0.009
Absent	68 (93.2%)	13 (68.4%)	
Present	5 (6.85%)	6 (31.6%)	

**Table 2:** Comparison of preoperative clinical imaging data between the STAS-negative group and STAS-positive group of the stage IA lung adenocarcinoma.

Variable	STAS negative (*N* = 73)	STAS positive (*N* = 19)	*P* value
Sex			0.549
Male	31 (42.5%)	6 (31.6%)	
Female	42 (57.5%)	13 (68.4%)	
Age	53.1 (10.9)	56.9 (7.61)	0.085
Maximum CT value (Hu)	-118.38 (141)	49.1 (62.9)	<0.001
Minimum CT value (Hu)	-553.00 [-659.00, -359.00]	-347.00 [-465.50, -203.00]	0.001
Mean CT value (Hu)	-321.60 [-442.01, -194.00]	-106.42 [-133.14, -60.51]	<0.001
Variance of CT values (Hu)	82.3 [58.4, 132]	115 [93.6, 152]	0.043
Kurtosis	2.40 [2.04, 2.50]	2.43 [2.13, 2.48]	0.732
Skewness	0.78 [0.39, 0.94]	-0.75 [-0.84, 0.65]	0.006
Maximum section area (mm^2^)	152 [87.6, 231]	336 [171, 408]	0.004
Superficial area (mm^2^)	679 [378, 1284]	1289 [852, 1921]	0.005
3D longest diameter (mm)	16.8 ± 6.01	25.3 ± 4.40	<0.001
Compactness	0.70 ± 0.17	0.61 ± 0.15	0.025
Sphericity	0.88 ± 0.08	0.84 ± 0.08	0.041
Entropy	8.19 [7.81, 8.57]	8.59 [8.38, 8.94]	<0.001
Location			0.659
Right upper lobe	26 (35.6%)	7 (36.8%)	
Right lower lobe	18 (24.7%)	4 (21.1%)	
Right middle lung	5 (6.85%)	0 (0.00%)	
Left upper lung	16 (21.9%)	7 (36.8%)	
Left lower lobe	8 (11.0%)	1 (5.26%)	
Volume (mm^3^)	1641 [703, 2997]	3476 [2345, 4167]	0.001
CTR	0.46 [0.41, 0.49]	0.50 [0.49, 0.64]	<0.001

## Data Availability

The data used to support the findings of this study are available from the corresponding author upon request.
